# Application value of PET/CT in monophasic primary sacral synovial sarcoma: a case report and review of literature

**DOI:** 10.3389/fonc.2023.1309123

**Published:** 2024-01-09

**Authors:** Mingyan Shao, Rong Xu, Wanling Qi, Zhehuang Luo, Fengxiang Liao, Sisi Fan

**Affiliations:** ^1^ Department of Nuclear Medicine, Jiangxi Provincial People’s Hospital, The First Affiliated Hospital of Nanchang Medical College, Nanchang, Jiangxi, China; ^2^ Department of Pathology, Jiangxi Provincial People’s Hospital, The First Affiliated Hospital of Nanchang Medical College, Nanchang, Jiangxi, China

**Keywords:** sacral synovial sarcoma, monophasic, CT, MRI, PET/CT

## Abstract

**Background:**

Synovial sarcoma is a malignant tumor of mesenchymal origin with a high degree of malignancy and easy metastasis. It mostly occurs in distal extremities or adjacent joints, and it is most common in deep knee joint. Primary sacral synovial sarcoma (PSSS) is extremely rare. The PET/CT imaging findings of a case of monophasic PSSS were reported. The clinical, imaging, and pathological data were summarized, and the literature was reviewed.

**Case description:**

A 67-year-old female patient presented with sacrococcygeal pain without obvious causes on 16 September 2022, with occasional pain at night, as well as aggravated pain during hip flexion and long-distance walking, which could be slightly relieved with rest, without special treatment. For further treatment before 1 month to Jiangxi Provincial People’s Hospital, after admission, laboratory tests were negative. Non-contrast CT scan showed expansive bone destruction in the S1-3 vertebrae with soft tissue density of about 58 mm × 46 mm × 52 mm. The boundary was clear, necrosis was visible within the vertebrae, and the boundary between the mass and the anterior sacral blood vessels and rectum was unclear. Non-contrast MRI scan showed mixed signals in lumbosacral masses, with equal signals in T1 and uneven and slightly higher signals in T2. Cystic degeneration and necrosis were visible, with multiple compartments in the lumbosacral masses. MRI enhancement showed uneven enhancement of lumbosacral mass with multiple compartments and no enhanced cystic lesion. The left sacral alar bone is destroyed, as shown by large flaky uneven strengthening. PET/CT showed that S1-3 vertebral body and left sacral alar bone were destroyed and soft tissue shadow formed, invading the sacral canal and the left foramina of S1-3. FDG metabolism was significantly increased, and malignant tumor was diagnosed by PET/CT. Pathological examination: The pathological diagnosis was monophasic PSSS. After systemic chemotherapy and local radiotherapy, no significant signs of recurrence and metastasis were found on CT so far. Follow-up treatment was continued.

**Conclusion:**

The incidence of PSSS is very low, its clinical and imaging manifestations lack characteristics, and the final diagnosis still needs pathology. PET/CT imaging has a certain value in the diagnosis of PSSS and has great application value in the preoperative staging, postoperative efficacy evaluation, and follow-up.

## Introduction

Synovial sarcoma (SS) is a mesenchymal origin malignant tumor with high malignancy, easy metastasis, difficult early diagnosis, and final diagnosis, which still requires pathology (1). SS mostly originates in the distal extremities or adjacent joints, and it is most common in the depth of the knee joint. Primary sacral synovial sarcoma (PSSS) is extremely rare (2). There are no obvious clinical symptoms in the early stage, as well as lumbosacral pain and nerve compression symptoms in the late stage. The imaging manifestations have no obvious characteristics and are mostly reported in individual cases. This paper reports the PET/CT imaging findings of a case of PSSS. The clinical imaging and pathological data of the case are summarized, and the related literature is reviewed in order to improve the understanding and diagnostic ability of the disease and to provide help for future patients.

## Case description

A 67-year-old female patient presented with sacrococcygeal pain without obvious causes on 16 September 2022, with occasional pain at night, as well as aggravated pain during hip flexion and long distance walking, which could be slightly relieved with rest, without special treatment. At the beginning of the disease, the patient’s spirit and diet were fine, sleep was normal, urine and bowel were normal, and there was no significant change in weight. For further treatment before 1 month to Jiangxi Provincial People’s Hospital, physical examination on admission shows the following: the sensation of left lateral ankle, left lateral calcaneus, and popliteal fossa decreased slightly; the muscle strength of left dorsal extensor and ankle plantar flexor muscle was grade 4; and the muscle strength of extensor toe long muscle was grade 3. Bilateral ankle reflexes were not elicited, straight leg elevation test was positive, and Thomas sign was positive. Laboratory tests were negative. Non-contrast CT scan (**Figure 1**) showed expansive bone destruction in the S1-3 vertebrae with soft tissue density of about 58 × mm 46 × mm 52 mm. The boundary was not clear, calcification and necrosis were visible within the vertebrae, and the boundary between the mass and the anterior sacral blood vessels and rectum was unclear. Non-contrast MRI scan (**Figure 2**) showed mixed signals in lumbosacral masses, with equal signals in T1 and uneven and slightly higher signals in T2. Cystic degeneration and necrosis were visible, with multiple compartments in the lumbosacral masses. MRI enhancement showed uneven enhancement of lumbosacral mass with multiple compartments and no enhanced cystic lesion. PET/CT (**Figure 3**) showed that S1-3 vertebral body and left sacral alar bone were destroyed and soft tissue shadow were formed, invading the sacral canal and the left foramina of S1-3, and there are no signs of local dissemination along sacral nerves. FDG metabolism was significantly increased, and malignant tumor was diagnosed by PET/CT. No clear metastasis was found in other parts. Because there was no obvious metastasis in the whole body and the preoperative diagnosis was not clear, surgical resection was given. hematoxylin-eosin (H-E) staining (**Figure 4**) showed that the epithelioid structure and sarcomatoid components could be seen under the microscope, the sarcomatoid components contained abundant spindle forming fibrocytes and increased interstitial blood vessels, and cystic necrosis areas could be seen, without calcification and ossification. Immunohistochemical markers of tumor cells are the following: A8: vimentin (+), CK (+, individual), TLE-1 (+), CD99 (+), CD10 (+), Desmin (+), H-Caldesmon (+), ER (+), PR (+, Part), Syn (+, Part), CD56 (+), CD21 (−), CgA (−), CD34 (−), CD31 (−), STAT6 (−), SOX-10 (−), S-100 (−), Bcl-2 (+, pulp), MUC4 (−), RB (+), CD45 (−), and Ki-67 (+, about 15%). *In situ* molecular hybridization: EBER (−). The pathological diagnosis was monophasic PSSS. The patient’s vital signs were stable after operation, and routine dressing change and fluid rehydration were used to prevent infection. After systemic chemotherapy and local radiotherapy, no significant signs of recurrence and metastasis were found on CT so far. Follow-up treatment was continued.

**Figure 1:** Female, 67 years old, primary sacral synovial sarcoma. **(A)** Axial CT. **(B)** Coronal CT. **(C)** Axial CT. **(D)** Sagittal CT. CT scan showed expansive bone destruction in the S1-3 vertebrae with soft tissue density of about 58 mm × 46 mm × 52 mm. The boundary was not clear, calcification (arrow, **A**) and necrosis (arrow, **B**) were visible within the vertebrae, and the boundary between the mass and the anterior sacral blood vessels and rectum was unclear.

**Figure 2:** Female, 67 years old, primary sacral synovial sarcoma. **(A)** T1-weighted images. **(B)** T2-weighted images. **(C)** Axial: T1 arterial stage 20s. **(D)** Sagittal: T1 arterial stage 20s. MRI plain scan showed mixed signals in lumbosacral masses, with equal signals in T1 (arrow, **A**) and uneven and slightly higher signals in T2. Cystic degeneration and necrosis were visible, with multiple compartments in the lumbosacral masses (arrow, **B**). MRI enhancement showed uneven enhancement of lumbosacral mass with multiple compartments and no enhanced cystic lesion (arrow, **C**).

**Figure 3:** Female, 67 years old, primary sacral synovial sarcoma. One hour after injection of 18F-FDG into PET/CT: **(A)** axial CT, **(B)** axial PET, **(C)** axial fusion, and **(D)** whole-body maximum intensity projection (MIP). PET/CT showed that S1-3 vertebral body and left sacral alar bone were destroyed and soft tissue shadow formed, invading the sacral canal and the left foramina of S1-3, necrosis and separation were visible within the mass, no significant FDG uptake was found in the necrotic area (arrow, **B**), FDG metabolism was significantly increased in the rest of the mass, and SUVmax was 4.9 (arrow, **C**).

**Figure 4:** Female, 67 years old, primary sacral synovial sarcoma. **(A)** H-E × 40, **(B)** H-E × 100, **(C)** H-E × 200, and **(D)** H-E × 400. H-E staining showed that the epithelioid structure and sarcomatoid components could be seen under the microscope, the sarcomatoid components contained abundant spindle forming fibrocytes and increased interstitial blood vessels, and cystic necrosis areas could be seen, without calcification and ossification.

## Discussion

Primary sacral synovial sarcoma (PSSS) is a rare mesenchymal origin malignant tumor. However, the origin of SS has nothing to do with synovial tissue, but it is called synovial sarcoma because the structure of tumor tissue is similar to synovial tissue under microscope (1). SS originates from the original mesenchymal stem cells around joints and tendons, and it is mostly found in the appendages of large joints of limbs, most of which are in the knee joint (3). SS generally grows slowly. It usually occurs in young adults, and the peak age of onset is 15–30 years old. There is no significant difference in incidence between men and women (4). This patient is 65 years old, which is higher than the age of onset reported in the literature. SS is clinically asymptomatic and usually presents as a deep painless mass, sometimes accompanied by local pain and tenderness, and occasionally severe pain (3). This case is a synovial sarcoma originating from the sacrum, which is very rare in clinic and has no characteristic clinical symptoms, mainly manifested as sacrococcygeal pain and left ankle numbness, and its symptoms are consistent with spinal compression of peripheral nerves and surrounding organs. Synovial sarcoma originates from undifferentiated mesenchymal cells, and it is a primary soft tissue malignant tumor characterized by bidirectional epithelial and stromal differentiation. The WHO New Classification of Soft Tissue Tumors (2013) classifies SS as malignant tumors with uncertain differentiation (5). Most synovial sarcomas are present in t (X;18) (p11.2;q11.2) chromosomal ectopia, generally thought to be caused by a chromosomal translocation between SS18 (SYT) on the long arm of chromosome 18 and SSX1, SSX2, or SSX4 on the short arm of chromosome X (6, 7). Pathologically, synovial sarcomas can be divided into monophasic fibrous, monophasic epithelial, biphasic, and poorly differentiated types according to the number and degree of differentiation of juvenile tumor cells, spindle tumor cells, and epithelioid cells in the tumor tissue (8). Typical synovial sarcomas appear on CT images as deep-seated soft tissue masses with a density equal to or slightly lower than the surrounding muscle, and a few have low densities similar to cysts. Calcification was seen in about 30% of the lesions, most of which were marginal calcification and showed patular appearance on CT images, whereas a few were extensive calcification or ossification (9). MRI can show equal signals on T1-weighted image (T1WI), equal height mixed signals on T2-weighted image (T2WI), and uneven enhancement of the mass. Jones et al. (10) first reported the typical manifestations of SS on MRI—”triplesign” in 1993, in which the tumor substance showed an equal signal; fresh bleeding and cystic necrosis showed a high signal; fibrocollagen, calcification, and old bleeding showed a low signal. The “paving stone” sign can be seen in the T2-weighted fat inhibition sequence, which is characterized by multiple nodules of varying sizes with slightly higher signal shadows accompanied by internal strips of lower signal separation (11). It has been reported that the imaging findings of SS have a certain correlation with pathological classification, and this case belongs to monophasic type. Due to the diversity of pathological components and differentiation degree, unipolar SS has both bidirectional and poorly differentiated MRI features (12). In this case, the signs of PSSS did not have these typical signs but showed a growth pattern of drilled holes, with a tendency to grow along the tendons, and synovium, cystic change, necrosis, and separation were seen inside. Most SS have variable or heterogeneous signals on T1WI or T2WI, and no clear imaging features have been used to distinguish paracral SS from other primary or metastatic neoplastic lesions (13). As a kind of functional metabolism imaging, PET/CT can diagnose the benign and malignant tumors through the metabolic information of ^18^F-FDG. PET/CT has the advantages of both CT and PET, which can display not only the sectional anatomical images but also the metabolic advantages of PET. Due to the high degree of malignancy of SS, the tumor is characterized by high metabolic activity. Due to internal capsular degeneration and necrosis, SS mostly showed heterogeneous mass increased FDG metabolism on ^18^F-FDGPET-CT. The median SUVmax of synovial sarcoma was 4.35, and the value ranged from 1.2 to 13.0, with a wide range. About 65% of primary synovial sarcoma had a SUVmax > 4.35 (14). The SUVmax of PSSS in this case was 4.9, which was consistent with literature reports. PSSS had a large metabolic overlap with other types of malignant tumors, resulting in the lack of obvious specificity of PET/CT in the diagnosis of SS. PSSS is highly malignant and prone to postoperative recurrence and metastasis. At present, the preferred treatment for PSSS is surgical resection, followed by adjuvant radiotherapy or chemotherapy (15). The 5-year and 10-year survival rates of SS are 83% and 75% in children and adolescents as well as 62% and 52% in adults, respectively. They are prone to local recurrence and metastasis in later stage (16). Therefore, PET/CT has great application value in preoperative staging, postoperative efficacy evaluation, and follow-up (17).

PSSS is rare and insidious in onset, painless, and slow in growth. Early diagnosis is difficult. With the enlargement of the lesion, it may cause pain and cause various symptoms and even seek treatment only due to sacral structure destruction, nerve root, and spinal cord compression, leading to spinal instability, vertebral collapse, and nervous system damage. This disease should be distinguished from common sacral tumors such as chordoma, giant cell tumor of bone, neurogenic tumors, and metastatic tumor. Chordoma on CT showed osteolytic destruction of the sacrococcygeal bone with some flaccid irregular calcification. Most tumors were accompanied by soft tissue masses. T1WI showed equal or slightly lower signals, T2WI showed higher or higher signals, and most tumors showed uneven signals. Giant cell tumor of bone presents with eccentric cystoid dilatant destruction of bone, mostly visible bony septa and bone ridge, forming a characteristic “soapy foam”–like sign, and may have intact or incomplete sclerotic edges. Extraosseous soft tissue mass is rare, and there is no calcification or ossification. Neurogenic tumors may be accompanied by partial enlargement of sacral foramen and intervertebral foramen, and the lesions involve both inside and outside the spinal canal. The typical lumps may present a “dumbbell” appearance, according to which they can be distinguished. Metastatic tumors often have a history of extracral tumors and are easily identified by PET/CT.

## Conclusions

In conclusion, PSSS is rare, and its clinical symptoms and radiographic findings are nonspecific. The diagnosis is determined by pathology, immunohistochemistry, and genetic testing. PET/CT has a certain diagnostic value in the diagnosis of synovial sarcoma. It combines the characteristics of functional imaging and anatomic imaging and is helpful for the clinical staging, therapeutic evaluation, and follow-up of PSSS.

## Data availability statement

The original contributions presented in the study are included in the article/supplementary material, further inquiries can be directed to the corresponding author/s.

## Ethics statement

Written informed consent was obtained from the individual(s) for the publication of any potentially identifiable images or data included in this article.

## Author contributions

MS: Conceptualization, Formal analysis, Writing – original draft, Writing – review & editing, Data curation. WQ: Conceptualization, Data curation, Writing – review & editing. RX: Conceptualization, Writing – review & editing. ZL: Conceptualization, Data curation, Writing – original draft. FL: Conceptualization, Data curation, Writing – original draft. SF: Data curation, Writing – review & editing.
